The article "Epipharynegal Abrasive Therapy Downregulates the Number of Epipharyngeal Abrasive CD4 Cells With Symptomatic Recovery" was published in 2023. Journal: Cureus.

# Epipharynegal Abrasive Therapy Downregulates the Number of Epipharyngeal Abrasive CD4 Cells With Symptomatic Recovery

**DOI:** 10.7759/cureus.50288

**Published:** 2023-12-10

**Authors:** Manabu Mogitate

**Affiliations:** 1 Otolaryngology, Mogitate ENT Clinic, Kawasaki, JPN

**Keywords:** nasopharynx, inflammation, epipharyngeal abrasive therapy, chronic epipharyngitis, cd4 (+) cell

## Abstract

Objective: In this study, the author focused on CD4 and CD8 profiles in epipharyngeal abrasive cells in patients with chronic epipharyngitis and investigated how the profiles differ from those in normal healthy subjects and how epipharyngeal abrasive therapy (EAT) influences these profiles.

Methods: This study included 18 patients (one male and 17 females, median age: 46 (30.0-56.5) years) who had been treated for chronic epipharyngitis between June 2021 and September 2021. Epipharyngeal abrasive cells were collected from patients with chronic epipharyngitis before EAT and three months after repeated EAT and were subjected to two-color flow cytometric analyses for CD4 and CD8 expression. The severity of participants’ symptoms was monitored using the visual analog scale.

Results: Symptoms of chronic epipharyngitis were significantly abated after three months of repeated EAT (p <0.001). The number of epipharyngeal abrasive CD4(+) T cells in patients with chronic epipharyngitis before EAT, which was significantly higher than that in normal healthy subjects (p <0.01), significantly decreased by the third month of repeated EAT (p = 0.01), alongside symptomatic recovery.

Conclusion: These results suggest that epipharyngeal CD4(+) T cells may have a critical role in treating the persistent inflammation of chronic epipharyngitis, and EAT may reduce the number of CD4 cells, which results in symptomatic recovery.

## Introduction

The epipharyngeal mucosa, an immunologically active site, functions as a source of immunoglobulin (Ig) A- and IgG-producing B cells [1]. Chronic epipharyngitis [2] not only presents local symptoms due to inflammation but also contributes to the development of systemic diseases via focal inflammation such as immunoglobulin A nephropathy, myalgic encephalomyelitis/chronic fatigue syndrome, and post-coronavirus disease (COVID) conditions [3-9]. Epipharyngeal abrasive therapy (EAT), a treatment option for chronic epipharyngitis, has been reported to improve not only local symptoms but also various systemic symptoms by suppressing inflammation in the epipharynx [10].

The epipharyngeal mucosa is mainly covered by a ciliated epithelium, which differs from those of the mesopharynx and hypopharynx, which are covered by a squamous epithelium. A number of lymphocytes containing predominantly B cells (about 65%), approximately 5% macrophages, and 30% CD3(+) T cells are mainly present in the submucosa. The T cells are primarily CD4(+), a subset (approximately 80%) [11]. In contrast, the surface mucosa of the epipharynx is rich in dendritic cells and CD4(+) T cells, some of which penetrate epithelial tight junctions and facilitate access to antigens.

The article "Epipharynegal Abrasive Therapy Downregulates the Number of Epipharyngeal Abrasive CD4 Cells With Symptomatic Recovery" was published in 2023. Journal: Cureus.

Nishi et al. [12] reported histologically that EAT causes squamous epithelialization of the epipharyngeal ciliated epithelium. As nitric oxide (NO) is produced in the ciliated epithelium [13], EAT may have reduced the pathological ciliated epithelium in the epipharynx, resulting in lower exhaled NO levels, as the author previously demonstrated [14, 15]. Nishi et al. [12] also reported that EAT suppressed the mRNA expression of interleukin (IL)-6 and tumor necrosis factor-alpha (TNF-α) in the submucosa of the epipharynx and had immunological efficacy. However, Hotta et al. [5] reported that many patients with IgA nephropathy, a tonsil-related and EAT-effect disease, have chronic epipharyngitis [6-8]. They also reported that CD4(+) T cells, especially CD4(+) human leukocyte antigen-DR isotype (HLA-DR)(+) cells representing activated helper T cells, in epipharyngeal abrasive cells that may originate from the surface mucosa of the epipharynx were significantly higher in patients with IgA nephropathy than in normal healthy subjects. Since then, there have been no reports examining the profiles of epipharyngeal abrasive cells in patients with chronic epipharyngitis or investigating how EAT influences the profiles of epipharyngeal abrasive cells.

In this study, the author focused on CD4 and CD8 profiles in the epipharyngeal abrasive cells of patients with chronic epipharyngitis and investigated how the profiles differ from those of cells in normal healthy subjects and how EAT influences these profiles.

## Materials and methods

Participants and setting

This study included 18 patients (one male and 17 females, median age: 46 (30.0, 56.5) years) who had been treated for chronic epipharyngitis between June 2021 and September 2021 and for whom epipharyngeal abrasive cells could be collected at the initial visit and three months after treatment. In addition, 18 normal, healthy subjects (six males and 12 females, median age: 36 (29.5-46.5) years) also participated. Patients’ data were collected retrospectively from medical records. The study was conducted per the principles of the Declaration of Helsinki and was approved by the Ethics Review Committee of Ota General Hospital, Kawasaki, Kanagawa, Japan (approval number: 22026).

Epipharyngeal abrasive therapy

At the initial examination, other organic diseases of the pharynx and larynx were excluded using an endoscope (endoscopy system: HOYA Corporation 2014, Tokyo, Japan; video processor: EPK-i7000, Pentax Medical, Tokyo, Japan; video transnasal scope: video naso-pharyngo-laryngoscope VNL-1190STK-1190STK, Pentax Medical). Normal white light was then used to diagnose chronic epipharyngitis. Patients’ epipharyngeal findings were assessed, and patients with bleeding during EAT were diagnosed with chronic epipharyngitis. Epipharyngeal abrasive therapy was performed once a week (one session) for three months using a transnasal and transoral approach in a blind fashion in principle. Endoscopic EAT was performed initially and then after the completion of 12 sessions.

The article "Epipharynegal Abrasive Therapy Downregulates the Number of Epipharyngeal Abrasive CD4 Cells With Symptomatic Recovery" was published in 2023. Journal: Cureus.

Epipharyngeal abraded cells

Epipharyngeal abrasive cells were collected orally with a disposable applicator before EAT during the treatment period. Before the initial endoscopic EAT and three months after treatment, the cotton portion of the applicator tip was cut off and inserted into a heparin-containing test tube (5 ml saline and Na 65IU heparin) for specimen submission, covered with a lid, and submitted to flow cytometric analyses in the subcontractor (SRL Ltd., Tokyo, Japan).

Two-color flow cytometry

Two-color immunofluorescence flow cytometry was performed using fluorescein isothiocyanate-conjugated anti-CD4 antibody (T4-FITC, Beckman Coulter, Brea, CA) and phytoerythrin-conjugated anti-CD8 antibody (T8-RDI, Beckman Coulter), which were reacted with abrasion cells for 20 min at 4°C. A lysing regent was added, mixed, and left for 10 minutes at room temperature. After centrifugal washing and removal of the supernatant, phosphate-buffered saline (PBS) was added, further centrifuged to remove the supernatant, and then measured via flow cytometry (BD FACSCanto II, Becton Dickinson Biosciences, Erembodegem, Belgium). The data were displayed as dot plots.

Symptom monitoring

Visual analog scale (VAS) scores (a VAS score of 10 indicates the worst symptom imaginable, and a score of 0 indicates no symptom) were used for monitoring symptom severity. Patients were asked to rate their symptoms (on a scale of one to 10) before EAT and three months after EAT.

Statistical analysis

The Mann-Whitney U test and the Wilcoxon signed-rank test (with Bonferroni correction) were performed on the results of flow cytometry of epipharyngeal abrasive cells in normal healthy subjects and patients with chronic epipharyngitis at the initial visit and after three months of treatment, respectively. All analyses were performed using IBM SPSS software version 22.0 (IBM Corp., Armonk, NY), with p <0.05 being considered statistically significant.

The article "Epipharynegal Abrasive Therapy Downregulates the Number of Epipharyngeal Abrasive CD4 Cells With Symptomatic Recovery" was published in 2023. Journal: Cureus.

## Results

The study included 18 patients (one male and 17 female) aged 15-67 years (median age: 46 (30.0-56.5) years) and 18 normal healthy subjects (six males and 12 females, median age: 36 (29.5-46.5) years). There was no significant difference in age and sex distribution between patients and normal healthy subjects (Table 1).

**Table 1:** Characteristics of the control group and the patients IQR: interquartile range

Control or patients		Control group	Patients
Number of materials		18	18
Age	Median	36	46
	IQR	(29.5-46.5)	(30.0-56.5)
Gender	Male	6	1
	Female	12	17

The main symptoms of the 18 patients were as follows: throat discomfort (seven cases), postnasal drip (three cases), nasal obstruction (two cases), sputum (two cases), nasal discharge, throat pain, fatigue, and IgA nephropathy (one case each). The VAS score of the chief symptoms significantly decreased after three months (12 times) of EAT (10 vs. 4.5 (3-6.5), p <0.01; Figure 1).

**Figure 1:** Symptom severity before epipharyngeal abrasive therapy (EAT) and three months after EAT Visual analog scale (VAS) scores (a VAS score of 10 indicates the worst symptom imaginable, and a score of 0 indicates no symptom) were used for monitoring symptom severity. The VAS score of the chief symptoms significantly decreased after three months of treatment (10 vs. 4.5 (3-6.5), p <0.01). The Wilcoxon signed-rank test was used for this analysis.

The results of two-color flow cytometry for epipharyngeal abrasive cells are shown in Table 2.

**Table 2:** Results of the two-color flow cytometric analysis of epipharyngeal abrasive cells in normal, healthy subjects and patients. The data were expressed as medians (interquartile ranges). The Man-Whitney U test (with Bonferroni correction) was used for this analysis.

CD4/CD8 profile	①Control	②Patients at the initial visit	③Patients after 3 months of EAT	p-value ①vs.②	p-value ②vs.③		
CD4(+)・CD8(−)	8.3 (3.3-11.0)	25.4 (13.4-30.6)	7.4 (4.6-14.3)			0.001	0.003
CD4(−)・CD8(+)	3.4 (1.5-9.3)	4.8 (3.9-14.9)	2.7 (2.1-3.3)			0.164	0.004
CD4(+)・CD8(+)	4.7 (4.0-20.5)	4.2 (2.4-4.8)	4.7 (3.2-10.3)			0.099	>0.999
CD4(−)・CD8(−)	74.9 (57.2-84.6)	61 (45.4-71.7)	80.7 (76.1-87.0)			0.068	0.013
CD4/CD8 ratio	1.9 (1.0-2.6)	3.1 (1.7-6.6)	2.5 (1.9-5.5)			0.038	0.089

There were significantly more epipharyngeal abrasive CD4(+) cells in patients with chronic epipharyngitis than in normal healthy subjects before EAT (25.4 (13.4-30.6) vs. 8.3 (3.3-11.0), p = 0.001). The CD4/CD8 ratio of epipharyngeal abrasive cells from patients with chronic epipharyngitis was significantly higher than that of the same cells from normal healthy subjects (2.0 (1.5-3.8) vs. 1.1 (1.0-1.5), p = 0.007). After three months (12 sessions) of EAT, the CD4 and CD8 profiles in epipharyngeal abrasive cells were similar to those of normal healthy subjects. The percentage of CD4(+) cells in epipharyngeal abrasive cells after three months of EAT significantly decreased as compared to that during the pretreatment period (7.4 (4.6-14.3) vs. 25.4 (13.4-30.6), p = 0.003).

The article "Epipharynegal Abrasive Therapy Downregulates the Number of Epipharyngeal Abrasive CD4 Cells With Symptomatic Recovery" was published in 2023. Journal: Cureus.

## Discussion

The organism is protected against inhaled foreign antigens by mucosal immunity, including that offered by the nasopharynx-associated lymphoid tissue [16]. In humans, the palatine tonsil and pharyngeal tonsil (adenoid), the largest components of Waldeyer’s tonsillar ring, are thought to play a central role [17]. During childhood, the pharyngeal tonsil (adenoid) is situated on the roof of the epipharynx, posterior to the nasal cavity. The adenoids start to shrink before adolescence, and then lymphoid follicles develop in the epipharyngeal submucosa, which contain predominantly B cells (about 65%), approximately 5% macrophages, and 30% CD3(+) T cells, primarily of the CD4(+) subset (about 80%) [1]. However, the surface mucosa of the epipharynx is lined with ciliated columnar epithelial cells mixed with a number of dendritic cells, macrophages, and CD4(+) T cells, just like lymphoepithelial lesions (LESs) of the palatine tonsil [18].

In this study, the CD4(+) T cells were significantly more detected on epipharyngeal abrasive cells, which may originate from the surface mucosa of the epipharynx, in patients with chronic epipharyngitis. Furthermore, the repeated EAT resulted in a significant decrease in the number of epipharyngeal abrasive CD4(+) T cells after three months, together with symptomatic recovery. These results suggest that epipharyngeal CD4(+) T cells may play a critical role in the persistent inflammation of chronic epipharyngitis, and EAT may reduce the number of CD4(+) T cells, resulting in symptomatic recovery. An increase in the number of CD4(+) epipharyngeal abrasive cells has also been reported by Hotta et al. [5], who demonstrated that the number of CD4(+) T cells, especially CD4(+) HLA-DR(+) cells representing activated helper T cells, in the epipharyngeal abrasive cells was significantly increased in patients with IgA nephropathy, which is one of the EAT-effective diseases. The CD4(+) CD25(+) T cells, i.e., activated helper T cells, are also reported to be more numerous in the tonsils of patients with pustulosis palmaris et plantaris [19], which is one of the EAT-effective diseases [6-8]. In addition, post-COVID conditions, which are also reported to be one of the EAT-effective diseases, are said to be characterized by increased numbers of peripheral blood CD4(+) T cells [20]. These reports support the involvement of epipharyngeal abrasive CD4(+) T cells in the pathogenesis of chronic epipharyngitis. Nishi et al. [12] microscopically demonstrated that EAT induces squamous metaplasia, resulting in the disappearance of ciliary structures of the surface mucosa of the epipharynx. The appearance of squamous epithelialization and submucosal fibrous stroma may physically inhibit the distribution of CD4(+) T cells to the mucosal epithelium.

The article "Epipharynegal Abrasive Therapy Downregulates the Number of Epipharyngeal Abrasive CD4 Cells With Symptomatic Recovery" was published in 2023. Journal: Cureus.

Although the pathogenic role of epipharyngeal abrasive CD4(+) T cells originating from the surface mucosa of the epipharynx has not been clarified in this study, it is speculated as follows: the CD4(+) T cells in the surface mucosa of the epipharynx may be activated by antigen-presenting cells in response to foreign antigens and invade the submucosa, resulting in the production of pro-inflammatory cytokines that activate other immune cells [21].

Nishi et al. [22] demonstrated that the mRNA expressions of IL-6 and TNF-α in B cells in the submucosa of the epipharynx increase in patients with chronic epipharyngitis, and EAT suppresses these expressions. It is possible, on the basis of these reports, that the CD4(+) T cells invading the submucosa from the surface mucosa may activate B cells expressing the mRNA of IL-6 and TNF-α, resulting in the secretion of such cytokines and leading to the development of symptoms and/or diseases caused by chronic epipharyngitis.

The limitations of this study include the small number of cases and the single-center study design. Therefore, it is recommended that the findings of this study be investigated further by multicenter studies in the future. The authors also did not assess changes over time in patients with chronic epipharyngitis who did not receive treatment; further investigation is needed to determine how EAT immunosuppresses CD4(+) T cells.

## Conclusions

Patients with chronic epipharyngitis have significantly more epipharyngeal abrasive CD4(+) T cells than normal healthy subjects. The number of epipharyngeal abrasive CD4(+) T cells significantly decreased by the end of three months of repeated EAT, together with symptomatic recovery. These data suggest that epipharyngeal CD4(+) T cells may play a critical role in the pathogenesis of the persistent inflammation of chronic epipharyngitis, and EAT may reduce the number of CD4 cells, resulting in symptomatic recovery.
